The article "Application of Image-Fusion 3D Printing Model in Total En Bloc Spondylectomy for Spinal Malignant Tumors" was published in 2022. Journal: J Healthc Eng.

# Application of Image-Fusion 3D Printing Model in Total En Bloc Spondylectomy for Spinal Malignant Tumors

**DOI:** 10.1155/2022/7907191

**Published:** 2022-08-31

**Authors:** Yushan Wang, Yi Xiang, Qiaoqiao Tian, Wei Luo, Hao Fan, Peng Ren, Zhi Lv, Jia Lv, Junjun Bai, Xiaochen Qiao, Yi Feng

**Affiliations:** ^1^Department of Orthopedics, The Second Affiliated Hospital of Shanxi Medical University, No. 382 of 51 Road, Taiyuan, Shanxi, China; ^2^Department of Orthpaedics, The Logistics Support Forces of Chinese PLA 985 Hospital, Taiyuan, Shanxi, China; ^3^School of Material, Taiyuan University of Technology, Taiyuan, Shanxi, China

## Abstract

**Purpose:**

To examine the effects of 3D printing model in total en bloc spondylectomy (TES).

**Methods:**

We performed a retrospective chart review of 41 cases of spinal tumors at our institution between 2017 and 2020, in which TES was applied. There were 19 cases with 3D printing model and 22 cases without 3D printing model. Operation time, intraoperative blood loss, excision range, complications, VAS, and ASIA grades were recorded. Statistical methods were used to analyze the data. KaplanMeier survival curve was made to evaluate the survival.

**Result:**

There were significant differences in intraoperative blood loss between the two groups. The rate of R0 resection and tumor envelope preservation were higher in 3D group than that in non-3D group. In 3D group, the complications included surgical site infection (5.2%) and cerebrospinal fluid leak (15.7%). In non-3D group, the complications included cerebrospinal fluid leak (27.3%) and nerve root injury (13.6%). The pain and neurological dysfunction were significantly relieved before and after surgery in 3D group. However, the neurological relief in non-3D group patients was not complete. The VAS scores of non-3D group at 6 months after surgery were much higher than that of 3D group.

**Conclusion:**

The application of 3D printing model not only helps surgeons observe the morphology, invasion range, and anatomic relationship of the tumor preoperatively, but also assists surgeons to judge, locate, and separate the tumor intraoperatively. For spinal malignancies, the 3D printing model is worth promoting.

## 1. Introduction

At present, the vast majority of spinal tumors are malignant. Spinal malignancies include primary and metastatic malignancies. Primary spinal malignancies are relatively rare in clinic, accounting for about 8–10% of bone tumors, while metastatic tumors are more common. With the progress of medical oncology in cancer treatment, the incidence of spinal metastatic tumors has been increasing year by year. And with the development of surgical techniques, more and more patients with spinal tumors have been benefiting from the surgical treatment, especially those with spinal malignancies. Total en bloc spondylectomy (TES) is an extra-lesional resection operation, which can not only reduce the local recurrence rate and prolong the survival of patients, but also significantly improve the quality of life. However, the anatomy of spine is complex. Tumors are often adjacent to important blood vessels, nerves, and organs, which makes TES difficult for surgeons. Traditional TES requires surgeons to have rich experience and spatial imagination ability, which are difficult to achieve. The key points of the operation are preoperative planning, intraoperative accuracy, and no postoperative complications. It is far from enough to rely on the preoperative imaging data such as X-ray, CT, and MRI. In recent years, the extensive application of 3D printing model in TES has helped the majority of doctors to solve many surgical problems. The 1 ∶ 1 made 3D printing models can clearly show the lesion and boundary, as well as the anatomic relationship with surrounding soft tissues, which is helpful to develop the best surgical plan and ensure the integrity and safety of tumor resection. In this study, we aim to evaluate the application effect of 3D printing model in TES.

The article "Application of Image-Fusion 3D Printing Model in Total En Bloc Spondylectomy for Spinal Malignant Tumors" was published in 2022. Journal: J Healthc Eng.

## 2. Method

### 2.1. The General Condition of Patients

We performed a retrospective chart review of all cases of spinal primary malignant tumors and metastases at our institution between 2017 and 2020, in which TES was applied (Tables 1 and 2). All surgeries were done by the same surgeon. A total of 41 patients with spinal malignancies were covered. Among them, 3D printing models were applied in 22 patients. One of the reasons 3D printing models were not used in these patients was that 3D printing technology was still in its infancy at that time. In addition, patients had full autonomy in deciding whether to construct 3D printing models before surgery. The reason why not all patients underwent this program every year was also its relatively high cost. So, patients were divided into the 3D-printing-model group (3D group) and the non-3D-printing-model group (non-3D group). The mean age was 55 ± 11 and 58 ± 14 years, respectively. In 3D group, there were 10 cases of spinal metastases and 9 cases of primary tumors. In non-3D group, there were 16 cases of spinal metastases and 6 cases of primary tumors. Except one patient, all the patients underwent one-stage posterior surgeries. For that patient, due to the large size, the tumor was removed by a combined anterior and posterior approach. All the patients received conventional radiotherapy and/or chemotherapy before and after surgery according to the nature of the tumor. The inclusion criteria were (1) patients with primary spinal tumors and metastatic tumors who underwent TES after evaluation by Tomita score and Enneking stage; (2) patients with local pain, neurological dysfunction, and other manifestations; (3) patients with complete clinical data; and (4) patients who gave informed consent to the treatment and research. Exclusion criteria were (1) patients with extensive metastasis; (2) patients who underwent non-TES surgeries; and (3) patients whose follow-up were lost.

The article "Application of Image-Fusion 3D Printing Model in Total En Bloc Spondylectomy for Spinal Malignant Tumors" was published in 2022. Journal: J Healthc Eng.

### 2.2. The Production of 3D Printing Model

Thin-layer CT, CTA, and MRI around the lesion were performed for all patients (Figures 1(a) and 1(b)). The layer thickness of CT was 1 mm and that of MRI was 1.5 mm. The FILES in Dicom format were imported into Mimics 17.0 software (Materialise, Belgium) and the 3D model was obtained by calculation. For tumors invading the spine canal and/or foramina, the 3D model would reveal the location of the patient's spinal cord and nerve roots, as well as their adjacent relationship to the tumor. For tumors that break through the anterior bone wall of the vertebral body, the 3D model would reveal the portion of the tumor which is located in front of the vertebral body, important blood vessels, and the relationship between them. It was worth noting that, compared with the 3D printing model relying solely on CT, the combination of CT and MRI could better display the actual scope of tumor invasion and its relationship with surrounding important structures, which would bring greater convenience to the surgeon (Figure 1). The rectification was completed by patching holes and removing highly-refracted edges in Geomagic 2014. The data was output to fused deposition modeling (FDM) 3D printers (Raise3d Pro2 Plus). The isometric model was made using poly lactic acid (PLA). According to the complexity of the model, the appropriate height, speed, support rate, filling rate, printing temperature were selected. The final 3D model was obtained after painting and coloring. The acquisition time was usually two days before surgery. The price of the model was around 3,000 yuan ($450).

### 2.3. The Formulation of Surgical Plan

The surgical approach (anterior, posterior, or combined) was determined by observing the anatomical relationship of the tumor. In non-3D group, the surgeon could only use two-dimensional images to infer the extent of tumor invasion and the anatomical relationship with surrounding structures. Therefore, the surgeon could only extrapolate what might happen during the procedure, the solution, and what to do with the implant roughly. In 3D group, the surgeon could clearly see the overall shape, size, and anatomical relationship of the tumor. Thus, during the simulation of intraoperative operations, the surgeon could clearly identify where delicate and careful operation was required and where was the “safe zone” for quick separation. In addition, some anatomic abnormalities and individual differences could be found at an early stage to rule out their influence on surgery. With the model, the length and the best site of the implant could be measured before the operation, thus saving the operation time and improving the operation efficiency.

The article "Application of Image-Fusion 3D Printing Model in Total En Bloc Spondylectomy for Spinal Malignant Tumors" was published in 2022. Journal: J Healthc Eng.

### 2.4. Surgical Procedure

The 3D model was displayed in a visible position at all times. After the laminas and spines around the lesion were exposed, the resection segments were determined according to the scope of the tumor and the pedicle screws were placed at the normal segments nearby. At this stage, the pedicles shown in the 3D model could assist in determining the angle of screw placement. Then, bilateral pedicles were sawed (or keep the side without tumor invasion). At this time, the position of the wire saw was adjusted by referring to the position of the nerve root in the 3D printing model to avoid nerve root damage. The lamina and spinous process were removed. After the spinal cord and the vertebral body were exposed, the dura mater and the nerve root should be carefully separated from the tumor tissues under the guidance of the 3D model. In this process, the 3D printing model was repeatedly observed to identify areas where the tumor was in close contact with the dura mater (and/or nerve roots). This model was clearly necessary to separate the tumor from the dura mater in front of the spinal cord. Because this operation could not be finished under direct vision during surgery. The integrity of the tumor envelope, dura mater, and the nerve root should be retained as far as possible. However, in non-3D group, the surgeon could only avoid the rupture of dura mater and the damage of nerve root by performing a slower and more careful separation. Moreover, the surgeon could only make careful and cautious attempts to separate the dura mater in front of the spinal cord under blind sight. For patients with tumor adhesion to the anterior blood vessels, the surgeon also needed to separate the anterior structures with the assistance of 3D printing models or under blind sight. After the separation, upper and lower discs of the diseased vertebra were cut off with an osteotome or a wire saw. Finally, the diseased vertebra together with the tumor was completely removed around the spinal cord, and the trimmed titanium mesh was placed for reconstruction (Figures 2(d)–2(f)). In 3D group, titanium mesh was based on a predetermined height in the model. But in non-3D group, the surgeon needed to prune the implant by measurement and repeated trials.

The article "Application of Image-Fusion 3D Printing Model in Total En Bloc Spondylectomy for Spinal Malignant Tumors" was published in 2022. Journal: J Healthc Eng.

### 2.5. Monitoring Indicators

The operation time, intraoperative blood loss, excision range, and complications were recorded. The resection range was divided into R0 resection and R1 resection. R0 resection means complete resection of the tumor and the resection margin is negative under the microscope. R1 resection means that the resection is complete under the naked eyes, but when viewed under the microscope, tumor cells can be seen at the margin. Pain levels before surgery, 1 week and 6 months after surgery were assessed by visual analogue score (VAS). Neurological function was assessed before and 6 months after surgery using ASIA grading. ASIA grading system is used to describe the damage degree of the neurological function. Grade A means the patient has no sensory and motor function below the damage level. Grade B means the patient has sensory function but no motor function below the damage level. Grade C means the patient has motor function, but the force of key muscles is below level 3. Grade D means the force of key muscles is above or equal to level 3. Grade E means the patient has normal sensory and motor function. The degree of the force of key muscles is divided into five levels. Level 0 means complete paralysis. Level 1 means the contraction of muscles can be touched. Level 2 means the patient can use the joint actively but cannot use it against gravity. Level 3 means the patient can use the joint actively against gravity. Level 4 means the patient can use the joint actively against moderate resistance. Level 5 means normality [1]. Kaplan-Meier survival curve was made to evaluate the survival of patients after TES.

### 2.6. Statistical Analysis

SPSS 25.0 software was used for statistical analysis. Quantitative data were expressed as the mean ± standard deviation, while qualitative data were expressed as the frequency. The chi square test or Fisher's exact test was used to compare the rates. The quantitative data were tested for normality before comparison. The data which obey normal distribution were analyzed using independent sample *T* test. The data which disobey normal distribution were analyzed using rank-sum test. *P* < 0.05 was considered statistically significant.

## 3. Result

TES was successfully completed in 41 patients. There were no significant differences in gender, age, and follow-up time between the two groups. In 3D group, the average operation time was 268 ± 62 min. The average blood loss was 1874 ± 1872 ml. In 5 patients, the integrity of the tumor envelope was damaged due to severe adhesion to the spinal cord or great vessels. Cerebrospinal fluid leakage occurred in 3 patients. Intentional nerve root sacrifice and vascular injury did not occur. Fifteen patients achieved R0 resection and four patients achieved R1 resection. Postoperative infection occurred in 1 case, and the incision healed completely after anti-infection treatment. In non-3D group, the average operation time was 286 ± 47 min, and the average blood loss was 2291 ± 716 ml. In 13 patients, the integrity of the tumor envelope was damaged due to severe adhesion to the spinal cord or great vessels. Cerebrospinal fluid leakage occurred in 6 patients. Inescapable nerve root damage due to tumor location and adhesion occurred in three cases. The right L2 nerve root was damaged intraoperatively in a patient with spinal metastases from breast cancer. Postoperatively, the patient presented with unilateral weakness of hip flexors. However, after 3 months, the symptom was significantly relieved. The other two patients also showed neurological impairment in varying degrees after surgery, but both achieved significant relief after a period of time. Twelve patients achieved R0 resection and ten patients achieved R1 resection. There was no infection at the surgical site in non-3D group (Table 2). There were no statistically significant differences in the operation time or the incidence of surgical complications between the two groups although the incidence of cerebrospinal fluid leakage and nerve root injury was significantly higher in the non-3D group than in the 3D group. After the application of 3D printing model, the probability of the envelope damage was significantly reduced. At the same time, the rate of R0 resection increased significantly. (*P* < 0.05) Postoperative X-ray films showed that all the lesions were removed in all patients, and the implants were in good position (Figure 2).

The article "Application of Image-Fusion 3D Printing Model in Total En Bloc Spondylectomy for Spinal Malignant Tumors" was published in 2022. Journal: J Healthc Eng.

In 3D group, the mean VAS was 6.1 ± 1.3 before surgery, 2.3 ± 0.9 one week after surgery, and 0.6 ± 0.7 six months after surgery. The pain levels of patients were significantly relieved before and after surgery (*P* < 0.05). Four patients were classified in Grade C, six in Grade D, and nine in grade E for ASIA grading before surgery. All but one patient (Grade D) were classified in grade E at 6 months postoperatively. The neurological function recovered significantly after TES (*P* < 0.05). Three patients had local recurrence during the follow-up period, two of whom died from the cancer and one of them underwent a second resection. To date, the patient has shown no recurrence. Of the 19 patients, six patients died including five who died from cancer-related complications and one who died from dyscrasia. Twelve patients remained tumor-free. Kaplan-Meier survival curve showed that the 3-year cancer-specific survival (CSS) rates in 3D group were 59% and the estimated median CSS time was 40.0 months (Figure 2). As for the implant, titanium mesh subsidence was found in 8 patients. The specific reasons need further research. In non-3D group, the mean VAS was 5.8 ± 1.2 before surgery, 2.2 ± 0.7 one week after surgery, and 1.6 ± 1.1 six months after surgery. The pain levels of patients were also significantly relieved before and after surgery (*P* < 0.05). One patient was classified in Grade B, one in Grade C, six in Grade D, and fourteen in grade E for ASIA grading before surgery. After TES, three patients were classified in Grade D and nineteen in grade E. There was no significant difference between preoperative and postoperative neurological function. Five patients had local recurrence during the follow-up period, four of whom died from the cancer and one of whom underwent a second resection without secondary recurrence. Of the 22 patients, nine patients died including eight who died from cancer-related complications and one who died from dyscrasia. Thirteen patients remained tumor-free. Kaplan-Meier survival curve showed that the 3-year cancer-specific survival (CSS) rates in 3D group were 48%, and the estimated median CSS time was 30.0 months (Figure 3). Titanium mesh subsidence was found in nine patients. There were no significant differences between the two groups in recurrence rate, oncologic outcome, preoperative and postoperative ASIA grades, titanium mesh subsidence rate, and VAS scores before and one week after surgery. However, VAS scores at 6 months after surgery were significantly higher in the non-3D group than in the 3D group (Table 3).

## 4. Discussion

### 4.1. Current Status of Surgical Treatment in Spinal Tumors

Surgical tumor removal has been performed more frequently for a series of cancer types in the recent decades despite the increasing efficacy of other modern systemic treatment modalities [2–6]. The importance of surgical treatment lies in its immediate effect on pain relief and nerve function recovery, which can greatly improve the quality of life and even prolong survival. In terms of surgical methods, piecemeal excision as a conventional surgery was commonly practiced. But its drawbacks were obvious. Because piecemeal excision is an intralesional removal, the presence of residual tumor cells may lead to incomplete symptom relief and recurrence in a short time. On this basis, TES has been applied more and more frequently. Since the vertebral body periosteum, anterior longitudinal ligament, ligamentum flavum, and to a lesser extend the posterior longitudinal ligament are considered barriers in the spread of vertebral tumors, an extra-lesional TES has been shown to result in superior oncologic outcome [7]. However, at the same time, the difficulty of the operation and the requirement of the operative experience are also quite high, which is the reason for high incidence rates of surgery related complications. Some researchers found that the complication rate was not charged by tumor extension or tumor etiology [7], indicating that the operator's subjective awareness played a decisive role in the outcome of the surgery. The difficulty of TES lies in the accurate cognition of tumor size and surrounding important anatomical structures. Conventional 2D imaging data, such as X-ray, CT, and MRI, cannot observe tumors in 3D perspective. It is difficult to know the real size and blood supply of tumors. Not to mention the relationship between tumors and important surrounding tissues. Thus, some problems arise, including massive bleeding, incomplete resection, long operation time, and so on. What's more, unexpected complications can occur, including nerve root damage, CSF leak, and even severe vascular injury, which will cause catastrophic consequences. Surgeons have focused on how to remove tumors safely and efficiently for a long time. Although 3D-reconstructed CT provides some help, the effect is limited because of insufficient display of soft tissues and the picture form of the result. Therefore, the need for a 3D model remains urgent.

The article "Application of Image-Fusion 3D Printing Model in Total En Bloc Spondylectomy for Spinal Malignant Tumors" was published in 2022. Journal: J Healthc Eng.

### 4.2. Application and Development of 3D Printing Technology in Spinal Surgery

In recent years, 3D printing technology has been widely used in clinic. In addition to the use of 3D printed anatomical models for preoperative planning and personalized guiding templates to improve the safety and success rate of pedicle screw placement, 3D printed customized implants and 3D bio-printing have also emerged [8]. Some researchers have found that titanium-alloy was designed with unique architectures based on 3D printing such as a highly interconnected and specific porous structure that mimics the architecture of trabecular bone, which can achieve better results of bone fusion [9, 10]. In addition, the combination of 3D printing with other technologies, such as finite element method, has also emerged to help surgeons better choose alternatives when a common screw-setting solution was difficult to achieve [11].

### 4.3. Advantages of 3D Printing Model for TES

At present, the biggest advantage of 3D printing technology in spine surgery is improving the accuracy of screw placement [12–15]. But for a spinal oncological surgeon, screw placement is often the easiest part of the procedure. Whether the size and location of the tumor can be accurately grasped and three-dimensional thinking are the most important determinants. 3D printing models play a critical role in the aspect. They can display the anatomical relationship of the lesion in a visual, three-dimensional, and comprehensive way. Surgeons can know the tumor morphology, invasive range, and the relationship with peripheral blood vessels and nerves intuitively, and then formulate a perfect surgical plan for tumor resection and stability reconstruction [16]. The prediction of the possible intraoperative situations will reduce the intraoperative possibility of artificial dissemination of tumor tissues and the incidences of complications, which will greatly shorten the operation time. As for the specific application of 3D printing model in TES, I think it is mainly in the following aspects. First, the presentation of the 3D printing model gives the surgeon an intuitive overall assessment of the tumor. This is a very important during operation. Because even if the surgeon carefully completed the preoperative planning, it is difficult to check all the details with the influence of other factors. At this time, the 3D printing model can be used as a prompt to give the surgeon some information about the anatomical relationship. When the surgeon disconnects the pedicle using T-SAW, especially for tumors involving the pedicle, the 3D printing model can help the surgeon locate the disconnection point and determine the path of adjacent nerve roots, thus avoiding the damage of tumor envelope and the nerve root. The 3D printing model can also provide the surgeon with a comprehensive and intuitive picture of the intra-canal invasion when the surgeon strips the tumor, which will help to achieve accurate and complete dissection. In addition, the role of 3D printing model is particularly important when the operation is in the blind area. For the tumor infiltrating the anterior spinal canal, the surgeon often separates the dura mater from the tumor blindly. At this point, the 3D printing model can provide an important guide to determine where the dissection should be careful and where the dissection is unnecessary. When the surgeon separates the affected vertebra, the 3D printing model can help the surgeon determine the separation plane to avoid breaking the tumor envelope. The 3D printing model can help to determine the distance between the anterior wall of the vertebral body and the blood vessels when spinning the affected vertebra out. It can also help to identify some special anatomy to avoid damage to the large blood vessels. According to the data, we found that there were almost no injuries to nerve roots or large vessels during surgery after the application of 3D printing model. However, 3 patients in the non-3D group experienced nerve root injury during surgery, which directly resulted in the worse outcome of postoperative neurological relief (Table 3). The rate of the complete preservation for tumor envelope in 3D group reached 73.7%, and R0 resection was completed in 84.2% of patients. But in non-3D group, the rate of the complete preservation for tumor envelope was 40.9%, and R0 resection was completed in 54.5% of patients. All the data showed that 3D printing models have greatly improved the accuracy of surgery. Therefore, the blood loss was less in 3D group, and the symptom relief was more complete. From the table, we found that residual cancer cells due to the destruction of the tumor envelope and incomplete resection might further lead to incomplete pain relief or recurrence of cancer pain in patients during long follow-up (6 months after TES). In other respects, preoperative design and measurement of implants can facilitate one-time reconstruction after tumor resection. What's more, in the process of doctor-patient communication, the application of 3D printing model can make it easier to explain the surgery, which is conducive to building a harmonious doctor-patient relationship.

The article "Application of Image-Fusion 3D Printing Model in Total En Bloc Spondylectomy for Spinal Malignant Tumors" was published in 2022. Journal: J Healthc Eng.

### 4.4. Current Shortcomings of 3D Printing Technology

Although the size of the model is consistent with the actual lesion, there may still be some differences, which may change the condition of the surgery. 3D printing models have also increased the length of stay and cost. With respect to the technology, the 3D printing technology cannot show the blood vessels' distribution of the tumor in detail. The realization of these possibilities depends on better technology and more complicated production process. But once achieved, the impetus for spinal tumor surgery will be profound.

## 5. Conclusion

The application of 3D printing model can help surgeons observe the morphology, invasion range and anatomic relationship of the tumor intuitively, which is useful to formulate a perfect surgical plan. During the operation, it can assist surgeons to judge, locate, and separate the tumor so as to achieve complete excision and symptom relief and reduce the incidences of complications. For spinal malignancies, the 3D printing model is worth promoting.

## Figures and Tables

**Figure 1:** (a) The extent of bone destruction and bone tumor invasion at each level was captured by CT and MRI. (b) The reconstructed 3D images were fused to show the anatomical relationships. The spinal cord was shown in yellow. The extent of tumor invasion was shown in red. The extent of bone destruction was shown in blue. (c) 3D images were printed into the PLA model. (d) Gross view of the tumor resected and postoperative X-rays.

The article "Application of Image-Fusion 3D Printing Model in Total En Bloc Spondylectomy for Spinal Malignant Tumors" was published in 2022. Journal: J Healthc Eng.

**Figure 2:** A 76-year-old male with chondrosarcoma diagnosed by needle biopsy. (a) MRI in the sagittal plane showed tumor invasion at T3, 4, and 5 levels. Transverse MRI showed that the tumor penetrated mainly to the left side of the vertebrae with left nerve root involved. The tumor showed low signal in T1 phase and medium high signal in T2 phase. (b) CT showed significant bone destruction. (c) The 3D printed model showed in detail the location and size of the tumor, the extent of its invasion in the bone tissue and its anatomic relationship with surrounding structures. (The tumor is in red). (d) The tumors completely removed during the operation were consistent with the 3D printed model in morphology, position, and other aspects. The capsule of the tumor was not destroyed. (e) On X-ray, we can see the gross structure of the lesion. The vertebrae and tumor were removed completely. (f) Postoperative X-ray showed complete removal of the lesion and good internal fixation. (g) Radiographs showed no local recurrence and solid internal fixation one year after surgery.

**Figure 3:** Cancer-specific survival (CSS) of 41 patients who underwent TES for malignant spinal tumor. In 3D group, the 3-year CSS rate after TES was 59% and estimated median CSS time after TES was 40.0 months. In non-3D group, the 3-year CSS rate after TES was 48% and estimated median CSS time after TES was 30.0 months. There was no statistical difference in survival time between the two groups (*P* > 0.05).

**Table 1:** General information of patients in 3D group.

Age (y)	Gender	Diagnosis	Area	Tomita score/Enneking stage	SA	OT (min)	BL (ml)	SSI	CSF leak	Doe	Rr	Tms	Recurrence	Os	VAS score			ASIA grade		FT (m)
															Pre	1w-po	6m-po	Pre	6m-po	
60	M	DL-BCL	T7	B5	Posterior	300	1500	−	−	+	R0	−	−	DOD	5	1	2	C	E	8
68	F	M	L2	3	Posterior	430	9000	−	−	+	R1	+	+	DOD	6	2	1	C	E	40
50	F	M	T5	5	Posterior	300	2000	−	−	+	R0	−	−	DOD	5	3	0	E	E	43
76	M	Chondrosarcoma	T3, 4, 5	B6	Posterior	260	1100	−	−	−	R0	+	−	NED	3	1	0	D	E	24
60	F	M	T11	5	Posterior	210	1300	−	+	−	R0	+	−	NED	7	3	1	E	E	32
56	M	Osteosarcoma	T3	B5	Posterior	240	800	−	−	−	R0	−	+	NED	5	2	1	E	E	24
63	M	M	C5, 6	4	Combined	390	2300	−	+	+	R1	−	−	NED	5	4	0	E	E	20
54	M	M	L2	3	Posterior	260	3500	−	−	−	R0	−	−	NED	6	3	1	D	E	18
48	F	M	T10	5	Posterior	220	900	−	−	−	R0	−	−	DOD	7	2	1	D	E	18
50	M	Plasmacytoma	T11	B5	Posterior	210	700	−	−	−	R0	−	−	NED	7	2	0	D	E	17
56	F	M	T7	5	Posterior	200	1000	−	+	−	R0	+	−	NED	7	3	1	E	E	16
26	F	M	T10	3	Posterior	230	2600	−	−	−	R1	−	−	NED	6	2	0	E	E	16
51	F	Plasmacytoma	T8	B5	Posterior	220	1000	−	−	−	R0	−	−	NED	7	3	0	C	E	15
73	F	Chondrosarcoma	L1	B4	Posterior	300	900	−	−	−	R0	+	+	DOD	5	2	0	E	E	9
57	M	CO	T3, 4, 5	B6	Posterior	330	2000	−	−	−	R0	+	−	NED	6	2	0	D	E	13
55	F	LL	L4	B5	Posterior	270	1500	+	−	−	R0	+	−	DOC	8	4	2	C	D	7
47	M	M	T3	5	Posterior	240	800	−	−	+	R0	−	−	NED	8	2	0	E	E	13
47	F	M	T12	5	Posterior	250	1500	−	−	−	R0	−	−	NED	5	1	1	E	E	12
53	F	Plasmacytoma	T11	B5	Posterior	230	1200	−	−	−	R0	+	−	NED	7	3	1	D	E	12

SA: surgical approach; OT: operation time; BL: blood loss; SSI: surgical site infection; CSF leak: cerebrospinal fluid leak; Doe: damage of envelope; Rr: resection range; Tms: titanium mesh subsidence; Os: oncology status; pre: preoperation; po: postoperation: 1w-po: 1 week postoperation; 6m-po: 6 months postoperation; combined: a combined anterior and posterior approach; DOC: death of cancer related complications; DOD: death of dyscrasia; NED: No Evidence of Disease; DL-BCL: Diffuse large B cell lymphoma; M: Metastatic tumors; CO: Chondroblastic osteosarcoma; LL: Lymphocytic leukemia.

The article "Application of Image-Fusion 3D Printing Model in Total En Bloc Spondylectomy for Spinal Malignant Tumors" was published in 2022. Journal: J Healthc Eng.

**Table 2:** General information of patients in non-3D group.

Age (y)	Gender	Diagnosis	Area	Tomita score/Enneking stage	SA	OT (min)	BL (ml)	SSI	CSF leak	Doe	Rr	Tms	Recurrence	Os	VAS score			ASIA grade		FT (m)
															Pre	1w-po	6m-po	Pre	6m-po	
56	M	Osteosarcoma	T3	B5	Posterior	400	2500	−	−	+	R0	−	−	NED	6	3	1	D	E	27
53	F	Plasmacytoma	T11	B5	Posterior	270	2500	−	−	+	R1	+	−	NED	4	2	0	E	E	36
48	M	M	T5	5	Posterior	280	2000	−	+		R1	−	+	DOC	7	3	3	D	E	9
74	M	M	L1	4	Posterior	330	3500	−	−	+	R0	−	−	NED	5	1	1	E	E	32
60	F	M	L3	2	Posterior	350	3000	−	+		R0	+	−	NED	5	2	1	E	E	25
51	M	Plasmacytoma	T11	B4	Posterior	270	1800	−	−		R0	−	−	NED	4	1	1	E	E	22
60	F	M	T8, 9	3	Posterior	340	3300	−	+	+	R1	+	−	NED	5	3	1	E	E	20
55	F	M	L3	5	Posterior	330	2700	−	−	+	R1	−	+	DOC	6	3	2	E	E	15
33	F	M	T8	2	Posterior	240	1200	−	−	+	R0	−	−	NED	5	2	2	E	E	28
66	M	M	T12	5	Posterior	270	1600	−	−		R1	+	−	DOC	7	3	2	D	E	22
63	F	M	T10	4	Posterior	240	1600	−	−	+	R1	−	−	DOD	6	2	2	D	E	8
62	M	M	L4	5	Posterior	330	3500	−	+	+	R1	−	−	NED	7	2	1	E	E	30
46	M	M	T12	5	Posterior	250	1600	−	−		R0	+	−	NED	5	3	2	E	E	33
51	F	M	L2	4	Posterior	320	2800	−	+	+	R1	+	−	DOC	5	2	1	E	E	30
74	F	M	T4	3	Posterior	230	1500	−	−		R0	+	−	DOC	7	2	2	E	E	16
20	M	Invasive GCTB	L2	B5	Posterior	260	2700	−	−	+	R0	−	−	NED	5	2	0	E	E	34
67	M	M	T11	5	Posterior	240	1800	−	−	+	R1	−	−	NED	8	3	2	B	D	28
70	M	M	T5	5	Posterior	220	1500	−	−		R0	−	+	DOC	5	2	3	D	E	11
80	F	Fibrosarcoma	L4	B5	Posterior	300	2900	−	+		R0	+	+	NED	4	1	1	C	D	18
67	M	M	L1	5	Posterior	270	2000	−	−	+	R0	−	−	DOC	7	2	1	E	E	30
56	F	M	T9	2	Posterior	250	1600	−	−		R0	−	−	NED	6	2	2	E	E	25
56	M	Chondrosarcoma	T3, 4	B6	Posterior	300	2800	−	−	+	R1	+	+	DOC	8	3	5	D	D	8

GCTB: giant cell tumor of bone.

The article "Application of Image-Fusion 3D Printing Model in Total En Bloc Spondylectomy for Spinal Malignant Tumors" was published in 2022. Journal: J Healthc Eng.

**Table 3:** Data statistics and analysis.

Factor	Condition	3D group	Non-3D group	
Gender	Male	8	12	
	Female	11	10	
Year		55 ± 11	58 ± 14	
Operation time (min)		268 ± 62	286 ± 47	

Blood loss (ml)		1874 ± 1872	2291 ± 716	*P* < 0.05

Complications	Surgical site infection	1 (5.2%)	0	
	Cerebrospinal fluid leak	3 (15.7%)	6 (27.3%)	
	Nerve root injury	0	3 (13.6%)	
Damage of envelope		5 (26.3%)	13 (59.1%)	*P* < 0.05

Resection range	R0	16 (84.2%)	12 (54.5%)	*P* < 0.05
	R1	3 (15.7%)	10 (45.5%)	

Titanium mesh subsidence		8 (42.1%)	9 (40.9%)	

Recurrence		3 (15.7%)	5 (22.7%)	

Oncological status	Death of dyscrasia	1 (5.2%)	1 (4.5%)	
	Death of complications	5 (26.3%)	8 (36.4%)	
	No evidence of disease	13 (68.4%)	13 (59.1%)	

VAS	Preoperation	6.1 ± 1.3	5.8 ± 1.2	
	1 week postoperation	2.3 ± 0.9 (*P*1 < 0.05)	2.2 ± 0.7 (*P*1 < 0.05)	
	6 months postoperation	0.6 ± 0.7(*P*2 < 0.05)	1.6 ± 1.1 (*P*2 < 0.05)	*P* < 0.05

ASIA	Preoperation	C : 4 D : 6 E : 9	B : 1 C : 1 D : 6 E : 14	
	Postoperation	D : 1 E : 18(*P*^*∗*^ < 0.05)	D : 3 E : 19	

Follow-up time (m)		19 ± 10	23 ± 9	

*P*1: the *P*1 value was obtained by comparing VAS scores before and 1 week after surgery. *P*2: the *P*2 value was obtained by comparing VAS scores 1 week and 6 months after surgery. *P*^*∗*^：the *P*^*∗*^ value was obtained by comparing ASIA grades before and 6 months after surgery.

## Data Availability

The data used to support the findings of this study are available from the corresponding author upon reasonable request.
